This article has been retracted.

# E-Health System Characteristics, Medical Performance, and Healthcare Quality at Jordan's Health Centers

**DOI:** 10.1155/2021/5887911

**Published:** 2021-11-26

**Authors:** Malik Bader Alazzam, Husam Al Khatib, Walid Theib Mohammad, Fawaz Alassery

**Affiliations:** ^1^Faculty of Computer Science and Informatics, Amman Arab University, Amman, Jordan; ^2^Al-Ahliyya Amman University, Amman, Jordan; ^3^Assistant Professor Organization Al-Hussein Bin Talal University, Princess Aisha Bint Al-Hussein Faculty of Nursing, Princess Aisha Nursing College Ma'an, Ma'an, Jordan; ^4^Department of Computer Engineering, College of Computers and Information Technology, Taif University, Taif, Saudi Arabia

## Abstract

This research explores how e-health systems' features (information quality, quality of the system, usability perceived, and perceived usefulness) contribute to improving medical personnel performance in medical centers, patient care, and physician-patient interactions in Jordan. The objective is to evaluate a single integrated model consisting of the technology acceptance model. This study used the logical research method and approach. A collection of data from 212 medical personnel working in 19 healthcare facilities throughout Jordan were gathered. To analyze the data collected and test the hypotheses of the research, a partially square/structural equation modeling method has been employed. The study found that the health information system (HIS) information quality has a direct and indirect beneficial effect on the performance of the staff, beneficial effects on patient care alone, and only favorable, indirect effects on the doctor-patient relationship. On the contrary, system quality was shown to influence directly and indirectly and to have a direct and indirect beneficial effect both on the connection between doctors and patients. Remember that the HIS has accessibility, speed, and mistake detection and avoids error issues. These shortcomings are suggested to be rectified in conjunction with improved user perception towards easy usage and utilization of the system.

## 1. Introduction

The use of technology is regarded as critical to the development of the health industry by many players in the health sector. Healthcare is a large and complex business, including interactions between stakeholders, leading to contradictory data and goals [1]. As a consequence, many nations are motivated by the use of new technology and advances in practice to modernize the health system. The current study in this area shows that the correct use of data systems significantly influences many essential people and organizational results. Information system (IS) offers timely and accurate users at all management levels information to promote improved efficiency, better planning, and better decision-making [2].

The importance of the use of IS and technology and the priceless benefits have attracted the interest of researchers and medical experts. This is because of globalization and the enormous advancements in medical technology. In the present difficult environment, information systems are intensively participated to maximize the performance of healthcare facilities in the healthcare sector [3]. In the present health application of the IS, a more sophisticated and intricate paradigm extends beyond the essential fulfillment of financial processes. IS has become a priority inside health organizations known as the health information system or e-health due to rapid and comprehensive medical technology advancements and increasing patient expectations. The potential for improving healthcare quality substantially and safety for patients is expected, improving the performance of personnel and clinics, reducing administrative medical mistakes, improving patient data access, improving clinical decision-making, and greatly reducing service cost [4–6].

Despite IS and HIS significant support and effects on organizational performance, current research indicates that IS and ERP systems are usually pricey and multifaceted and may provide unsatisfactory outcomes. Despite the success of many e-health systems and the profitability and well-being of implementing organizations, many other systems failed to fulfill their objectives. They even contributed to the deterioration in healthcare performance. Although companies have made extraordinary expenditures in the procurement of bespoke e-health systems in addition to developing them in-house, there really is no rigorous proof of effectiveness or profitability in the literature. Therefore, health organizations must examine if these systems adequately meet their operational requirements and enhance medical performance or health service [7].

Domínguez-Mayo et al. [8] studied the single integrated model covering D&M and IS user satisfaction/use in health settings. Integrating multiple IS models helps to improve the understanding of the effect of technology on complex environmental environments, in particular [9–13]. Such integration is thus often regarded as a positive practice that values our knowledge and understanding of IS adoption, acceptability, usage, and success. Their research also examined the near and distant determinants of system usage and user satisfaction, expressed in user performance, healthcare quality, and interactions between the physician and patient. Häyrinen et al. [14] stressed the need better to understand the variables influencing system resistance and user acceptance. Xu et al., Heo and Han, and Hidayah et al. [15–17] also stated that there is a need for more research to study the factors behind the variation in IS subjective norms. Hsu et al. [18] stated that the present study reveals combined findings with clinical outcomes on the association of e-health systems [19]. The present study is an effort to present research aimed at the impact of the e-health system on the clinical staff performance, patient care, and patient-doctor relationship using Jordan's population. There are no studies and research on IS theories and frameworks in the area [20–23].

## 2. Objectives

In reaction, the research focuses on the degree to which the newly introduced e-health system in Jordan affects clinical staff performance, patient care, and doctor-patient interaction. The remainder of this paper will concentrate on the following questions. The e-health system is created in-house as specific purpose software to meet clinician requirements and adapt to how the healthcare sector does everyday duties and activities. The system is regularly modified. The research takes doctor-patient relationships as another structure that should be affected by the use of e-health systems. The following objective statements represent the research objectives:

- To investigate the impact of the e-health system on the clinical staff performance, patient care, and doctor-patient interaction

The following two parts concentrate on the theoretical foundation, literary evaluation, study framework, and hypothesis formulation. The following section covers the many elements of the approach chosen. The paper then proceeds with data analysis and findings. The final three parts describe significant results, limits, theory, and practice reflection and pave the path for future study [24–26].

### 2.1. Literature Review

#### 2.1.1. Information Quality (IQ)

[27] IQ is defined as the intended functionality and utility of user IS output. Informational characteristics include timeliness, format, scope, correctness, consistency, usability, accessibility, usability adequacy, briefness, dependability, and relevance. Comparably, [28] IQ range expanded to evaluate the IS production or current and was the most often used to evaluate the quality of the information in its many elements, comprehensiveness, and accuracy. In addition, Salih and Ghazi Atiya [29] submitted that IQ provided a key predictor of end-user happiness and productivity results and described it as the content and structure of the output of the system to guarantee it is useful, adequately comprehensive, relevant, readable, and simple to comprehend. Patient interaction information with healthcare professionals must be of use in supporting physician and management choices [30]. The right and higher information is vital not only for providing high-quality clinical treatment but also for ongoing healthcare, sustaining the highest standards of healthcare, and economic and medical services' research, as well as healthcare system planning and administration [31].

#### 2.1.2. System Quality (SQ)

[32] The system quality is defined as the desired features of an information system emphasizing usability or performance measurements. Accessibility, sophistication, effectiveness, comfort, customization, accurate information and currencies, clarity of learning and utilization, versatility, integration, interaction, searching, dependability, responsiveness, system correctness, system features, and reversal time are all considered elements. Specifically, Abdulsattar Abdullah et al. [33] identified the system quality as an information system factor in the success of an information management system evaluating the information system and its characteristics, such as simplicity of use, ease of training, and usage. The user experience of a system was defined by Thanoon [34] in a different way than it has been described before from a technological, architectural, and operational standpoint. When the user evaluates system features such as ease of use, reliability, and response times, the user's perception of the system is reinforced. To assess SQ, Rodrigues et al. [35] focused on dependability, reliability, time response, and integration. They also supported the convenience, privacy, and fast response afforded by high levels of SQ. The qualities of response and learning are said to have the largest impact on the user content out of all of the variables examined [36].

#### 2.1.3. User Performance (UP)

Because of the nature and complexity of the services given to beneficiaries, the performance of healthcare workers and doctors became a significant concern. Thus, healthcare workers' responsibilities are essential to the daily well-being of the individual and must be provided professionally and organically. Due to fast technology propagation, during IS adoption, businesses invest a lot of money on automating, redefining, and reorganizing operations and business processes to increase personal and company performance, productivity, and efficiency.

Performance was based on the possible chance to perform specified activities to accomplish targets in the given time frame and limitations of the stakeholders and the circumstance [37]. The actual outcomes obtained contrasted with planned goals is another definition of performance. Several researchers, including [38], examined the extent to which various components of the system accomplish their primary goals. The functioning as described by Haux et al. [23] was to accomplish quantifiable targets, resulting from proper conduct and efficient use of the necessary knowledge, abilities, and skills. Consequently, work outcomes may be used to define performance since they have the greatest relationship to strategic organizational goals, customer satisfaction, and economic contributions, among other things. The previous definitions make it very apparent that performance refers to the extent to which intended objectives have been achieved [39].

#### 2.1.4. Patient Care (PC)

The advent of e-health systems and instruments has provided patients with new possibilities to be more engaged in their treatment and new options for high-quality and efficient patient care. Unless apparent advantages and a real added value exist, clinics will not be convinced to adopt e-health systems. The main advantage of e-health has been its contribution to better patient care. The importance of an excellent HIS in terms of high quality and effective patient care is clear since no effective treatment choices can be made without adequate access to the necessary patient data, which would have deadly implications for patient care.

#### 2.1.5. Doctor-Patient Relationship (DPR)

The significant development of healthcare technology has impacted the doctor-patient relationship intensely. This connection is important to the identification and recruitment of a successful disease plan by doctors and to patients' understanding of the nature and effects of the condition, participation in the treatment choice, and adherence to the doctor's recommendations.

### 2.2. Theoretical Framework

The health information system is the political and social solution that integrates all subsystems inside a medical setting and combines real actors in their different responsibilities in information processing with the use of technology. There are many different e-health versions, including electronic health records, hospital IS, computerized medical order entry, electronic prescription, bar-coded medicines' administration, and clinical decision support. There are also many different versions of e-health.

In spite of the major advances in methods and theories, the implementation of IS systems and solutions in particular and e-health systems is facing continuing difficulties for a long time. Aside from this, the development of information systems and e-health systems, in general, is costly and needs substantial expenditures. As a result, managers and shareholders are worried about whether an investment in information technology (IT) would enhance the performance of their companies. Management must consider the many aspects in order to maximize the return on their information technology investment via increased efficiency, effectiveness, and performance.

Given various IS stakeholder groups that have their own success criteria, a comprehensive model has become mandatory covering significant characteristics of success. Influence of how individuals perceive and create information systems' acceptance, usage, and satisfaction is very essential for system developers and organizations. This knowledge may assist companies in making better use of new technologies that are being developed.

The technology acceptance model is amongst the most common IS models used to explain how people accept and use technology. It has thus been overwhelmingly backed as a primary model in the study of acceptance and use of electronic health systems originally developed who have a strong theoretical background; and a considerable number of research studies have been used in various areas of studies for more than 30 years in a variety of contexts. The perceived usefulness of this model and the perceived simplicity with which it can be used are the two most important factors that affect IT adoption, end-user satisfaction, and the exact use of the system. The external variable, which can be social and religious factors, affects both constructs.

## 3. Methodology

The present study utilizes a deductive approach and quantitative technique and a positivist philosophy of research.  Figure 1 shows the effective TAM and IS models, based on the exact assumption of causal interconnections here between variables assessed via representative data, which are based on the primary research issue and the discussions in the previous paragraphs [40–42]. The research objective is to explain how e-health systems affect the clinical performance of staff, patient care, and doctor-patient relationship using the TAM and then D&M model (e-health system features) which influence results' variables (efficiency of medical personnel, patient care, and doctor-patient relationships). The positive method has been developed in the IS study and can forecast IS success by identifying the patterns of connections between causes and effects. In addition, the positive and quantitative methods are highly efficient in anticipating the hidden pattern of IS creation and success, as well as use, and evaluating user behavior and examining attitudes about the system are all important considerations [43].

This study utilizes the quantitative explanatory method in order to survey the target sample following its primary research question because it is one of the most successful instruments of IS research.

### 3.1. Sample and Population

At the moment, the topic of e-health is applied in Jordan's healthcare sectors. The population has been chosen as medical personnel (doctors and management), individuals who have previously made use of the technology and have developed opinions regarding its operation and effect on routine clinic activities. Extensive study indicates that medical personnel are a major stakeholder group that can acquire a better sense for the success and efficiency of e-health systems.

## 4. Results

### 4.1. Demographics of the Study

Demographics of the respondents are given in Table 1. The table shows the percentage distribution of the respondents by gender, marital status, age groups, qualification, and experience. Male and female respondents are seen in 71% and 29%, respectively, while 56.1% and 43.9% of the total populated response are single and married caressingly, which illustrates that most of the respondents are not married. Rest of the categorical distribution can be seen in the table.

### 4.2. Descriptive Statistics

Descriptive statistics for the study variables are given in Figure 2 and Table 2, which shows the number of populations, minimum, maximum, mean, and standard deviations. The descriptive analysis is a mean of presenting the summary of the variables. Table 2 shows the mean values of 2.40, 2.41, 2.37, 2.49, and 2.39 for information quality, system quality, user performance, patient care, and doctor-patient relationship, respectively.

### 4.3. Normality and Factor Analysis

Factor analysis shows a good result higher than 0.70 which suggests that components of the variables have excellent coherence and can be used in correlation and regression analyses (Table 3). KMO test was performed, and values of Cronbach's alpha were investigated which were 0.79, suggesting that the data are reliable to be used in the correlation and regression analysis.

### 4.4. Correlations

Correlation analysis was performed which shows a direct relationship, with a significance of *p* < 0.05. Information and system quality are directly proportional to user performance, patient care, and doctor-patient relationships (Table 4).

### 4.5. Regression Analysis

Regression analysis is used to investigate the impact of e-health on the clinician's user performance, patient care, and doctor-patient relationships. The results of the study show a significant positive impact of information quality on all of regressed variables as reported in Table 5.

However, using system quality as the predictor, the impact is also directly proportioned and significant at *p* < 0.05. On the contrary, the user performance impact is negatively significant.

## 5. Discussion

These findings indicate that IQ has a favorable effect on the (Table 6) performance of clinicians in health facilities. This supports the notion that an eye on the quality of information entered through into the e-health system leads to an improvement in the performance of clinical personnel. The developed the system's patient information quality, the greater the number of people that perceive and find it simpler to utilize and the more likely they intend to use the system and enhance its performance. These findings are consistent with prior research [44].

The awareness of clinicians that a developed system is easy to use and that it will help to easily fulfill their tasks assigned with their awareness of the system's capabilities. In contrast, the real SQ difficulties of system users such as frequent disconnection, system slowness, system confidence problems and data insertion mistakes, or the generation of outputs virtually cancelled the PF-mediated impact. This is consistent, which found that the performance and productivity of medical personnel had negative effects as a consequence of problems relating to reaction time, dependability, and input size limits for the system examined [45].

## 6. Conclusions

The research was aimed on the impact of e-health systems on the clinical staff performance, patient care, and doctor-patient relationship using the information system models. The followed study used collected primary data from Jordan's hospitals, and multilinear analysis examined the effect of e-health systems on doctoral relations, patient care, and user performance. This study was performed. The research found a substantial direct effect of the e-health system on the dependent variables [37]. The research found that information on patient engagement with healthcare providers could be useful for supporting physicians and treatment choices. These are helpful if they are accurate, useful, structured, and simple to use. Accurate and current information is required not just for high-quality clinical treatment but also for current healthcare and business research, as well as the creation and administration of healthcare delivery systems.

The study recognized SQ and IQ as IS success elements, which included assessing the information systems and their characteristics, such as ease of use, training, and system usability. The system was described as a user experience in a new way [4]. Users' opinions on system characteristics such as simplicity of use, dependability, and reaction times are influenced by their personal experiences [16].

## Figures and Tables

**Figure 1:** Conceptual framework of the study.

**Figure 2:** Gender distribution.

**Table 1:** Percentage distribution.

Table, *N* (%)		
Gender of the respondents	Male	71.0%
	Female	29.0%

Marital status of the respondents	Single	56.1%
	Married	43.9%

Age of the respondents	18–25 years	29.8%
	25–35 years	53.4%
	35–50 years	16.8%
	Above 50 years	0.0%

Qualification of the respondents	Graduation	40.2%
	Master	39.9%
	PhD	1.5%
	Others	18.4%

**Table 2:** Descriptive analysis of the variables.

	*N*	Minimum	Maximum	Mean	Std. deviation
Information quality	212	1.00	4.67	2.4072	0.94798
System quality	212	1.00	4.67	2.4104	0.93936
User performance	212	1.00	4.67	2.3742	0.90135
Patient care	212	1.00	5.00	2.4921	1.08387
Doctor-patient relationship	212	1.00	4.67	2.3915	0.92207
Valid *N* (listwise)	212				

**Table 3:** Reliability, factor, and normality analysis.

	Factor loadings	Normality (skewness)	Cronbach's alpha
Information quality	0.994	0.561	0.79
System quality	0.976	0.48	
User performance	0.922	0.627	
Patient care	0.937	0.482	
Doctor-patient relationship	0.987	0.499	

**Table 4:** Correlation analysis.

	Information quality	System quality	User performance	Patient care	Doctor-patient relationship
Information quality	1				
System quality	0.969^*∗∗*^				
User performance	0.905^*∗∗*^	0.868^*∗∗*^			
Patient care	0.924^*∗∗*^	0.897^*∗∗*^	0.785^*∗∗*^		
Doctor-patient relationship	0.988^*∗∗*^	0.967^*∗∗*^	0.887^*∗∗*^	0.910^*∗∗*^	1

^∗∗^Correlation analysis and significance of 0.5.

**Table 5:** Regression analysis.

	Information quality				
	*B*	Std. error	Beta	*t*	Sig.
User performance	0.994	0.112	1.045	8.842	0
Patient care	0.255	0.122	0.897	8.408	0
Doctoral-patient relationship	0.808	0.041	0.831	19.884	0

**Table 6:** Regression analysis.

	System quality				
	*B*	Std. error	Beta	*t*	Sig.
User performance	−0.139	0.113	−0.145	1.226	0.001
Patient care	0.320	0.123	0.028	0.263	0.003
Doctoral-patient relationship	0.159	0.041	0.162	3.877	0.000

## Data Availability

The data underlying the results presented in this study are available within the manuscript.
